# The crucial role of SRPK1 in IGF-1-induced EMT of human gastric cancer

**DOI:** 10.18632/oncotarget.20048

**Published:** 2017-08-07

**Authors:** Hong Wang, Chunlei Wang, Wenling Tian, Yanfen Yao

**Affiliations:** ^1^ Department of General Surgery, Shandong Provincial Third Hospital, Jinan, Shandong, China; ^2^ Thyroid Disease Prevention and Control Center, Shandong Provincial Institute of Endemic Disease Control, Jinan, Shandong, China; ^3^ Department of Intensive Care Unit, Shandong Provincial Third Hospital, Jinan, Shandong, China

**Keywords:** SRPK1, IGF-1, EMT, GC

## Abstract

In recent years, the insulin-like growth factor (IGF-1) and serine-arginine protein kinase 1 (SRPK1) have been reported to be implicated in the pithelial-mesenchymal transition (EMT) in many kinds of malignancies. However, the potential roles of IGF-1-SRPK1 signaling in the EMT of gastric cancer (GC) have not been investigated. In the present study, the in-vitro assays were used to investigate the molecular role of SRPK1 in cell cycle, motility and invasiveness. We demonstrated that the expressions of SRPK1 or insulin-like growth factor receptor 1 (IGF1R) were significantly increased in GC tissues and cells than those in normal tissues and GES-1 cells, and closely associated with metastasis, stage and prognosis. Western blot analysis showed that IGF-1 treatment can induce the expression of p-AKT and EMT biomarkers (N-cadherin, MMP2 and Slug) in a dose-dependent fashion in MGC803 and BGC823 cells. On the other hand, the knockdown of SRPK1 attenuated IGF-1-induced increase of EMT biomarkers and p-AKT. Besides, in-vitro analysis showed that knockdown of SRPK1 induced cell cycle arrest in G0/G1 phase, and affected cell migration and invasion. In conclusion, IGF-1-IGF1R pathway induced the expression of SRPK1 to control the progression of EMT via AKT pathway in the development of GC. Our findings lay a promising foundation for the IGF-1-IGF1R axis-targeting therapy in GC patients.

## INTRODUCTION

Gastric cancer (GC) is one of the most common solid malignant tumors [1]. Because locally advanced GC has high a frequency of micrometastasis and relapse, its prognosis is poor. The 5 years’ survival after radical surgery was 30%∼50%. Perioperative and adjuvant chemotherapy have been shown to be able to decrease distant metastasis and improve survival by 10–15% [2–4]. Chemoresistance likely has contributed to the relapse after chemotherapy. It is crucial to understand the underlying mechanism of chemoresistance and find novel therapeutic targets to further improve the outcome of GC.

The IGF1R is a transmembrane receptor tyrosine kinase, closely related to the insulin receptor (InsR) that forms homodimers or heterodimerizes with InsR to recognize its ligands, IGF-1 and IGF-2 [5]. Upon ligand binding, IGF1R activates multiple downstream signaling cascades, the two most prominent being PI3K/AKT and RAS/RAF/MEK/ERK [6]. PI3K/AKT enhances cellular metabolism and protein synthesis via mTOR and enhances survival via BAD/Bcl2, p53, NF-κB, and FOXOs, whereas RAS/RAF/MEK/ERK activation generally results in increased cellular proliferation [7]. In addition, SRPK1 was involved in regulating some mRNA-processing signalings, involving alternative splicing [8–10]. It has been reported that SRPK1 was highly expressed in many kinds of cancers, such as prostate cancer, breast cancer, lung cancer, and glioma [11]. A couple of reports demonstrated that inhibition of SRPK1 exerts anti-tumour effects on different tumors, therefore SRPK1 has become recommended as a novel candidate for cancer patient therapies [12, 13].

However, some molecular mechanisms underlying IGF1R/SRPK1-induced gastric cancer are not unraveled. To date, the potential action of IGF-1-SRPK1 pathway in the involvement of EMT of GC has not been reported. In the present study, the in-vitro assays were used to investigate the potential value of SRPK1. Our data confirmed a newIGF-1-SRPK1pathway involved in the EMT, which can be targeted to treat GC patients.

## RESULTS

### Expression of SRPK1 and IGF1R in gastric cancer tissues

To explore the role of SRPK1-IGF1R-EMT axis in the development of gastric cancer, we carried out the immunohistochemistry assay to analyze the expression of SRPK1 and IGF1R in 90 gastric cancer tissues. We found that five cases of gastric cancer samples showed a higher expression of SRPK1, with the expression rate of 83.3% (Figure 1A). On the other hand, the staining of SRPK1 was scarcely found in adjacent normal gastric tissues (Figure 1B). Additionally, 78 gastric cancer samples showed high expression of IGF1R, with the expression ratio of 86.7% (Figure 1C). We further observed that IGF1R expression was very low in adjacent normal gastric tissues (Figure 1D). According to Spearman's correlation analysis, we demonstrated that high expression of SRPK1 was obviously correlated to IGF1R expression in gastric cancer tissues (r = 0.912, *p* = 0.001).

**Figure 1:** Expression status of SRPK1 and IGF1R protein in gastric cancer tissues Immunohistochemical staining was conducted in all 90 gastric cancer tissue sections using anti-SRPK1 or anti-IGF1R antibodies, at the same time, the representative image was showed. SRPK1 (**A**, **B**) and IGF1R (**C**, **D**) protein showed different expression intensities (+∼+++, −).

### SRPK1, IGF1R expression and clinicopathology

Subsequently, we analyze the relationship between SRPK1/IGF1R expression and clinicopathology. We found that the expression of SRPK1 or IGF1R was not correlated to age or gender, and SRPK1 or IGF1R expression was closely correlated to histological differentiation (*p* = 0.018, *p* = 0.001), lymph node metastasis (*p* < 0.001, *p* = 0.016) and UICC stage (*p* < 0.000, *p* = 0.037) (Table 1).

**Table 1:** SRPK1 and IGF1R with clinicopathological indicators

Indicators	N	SRPK1		*p* value	IGF1R		*p* value
		High	Low		High	Low	
Age							
< 56	45	38	7	0.777	38	7	0.535
≥ 56	45	37	8		40	5	
Gender							
male	60	51	9	0.549	50	10	0.188
female	30	24	6		28	2	
Tumor size							
< 5 cm	65	55	10	0.091	60	5	0.011
≥ 5 cm	25	23	2		18	7	
Histology							
Well/moderate	59	46	13	0.018	45	14	0.001
Poor	31	30	1		30	1	
LN metastasis							
Yes	51	49	2	0.000	48	3	0.016
No	39	26	13		30	9	
UICC stage							
I-II	29	17	12	0.000	22	7	0.037
III-IV	61	58	3		56	5	

### SRPK1, IGF1R expression and prognosis

In the present work, we applied Kaplan-Meier curve to analyze the prognosis of gastric cancer patients. As shown in Table 2 and Figure 2, we found high and low SRPK1 expression group had a significant difference in overall survival. In addition, an obvious overall survival difference between high and low IGF1R expression group was also found. Statistically, our data revealed five years overall survival rate of in high SRPK1 group was 23.9%, and that in high IGF1R group was 25.1%. Furthermore, according to log-rank test analysis, we found that high SRPK1 or IGF1R expression was closely correlated with poor overall survival (*p* = 0.007, *p* = 0.037, respectively). At last, we carried out the univariate and multivariate analyses using Cox's proportional hazards regression model, and found that SRPK1 or IGF1R expression can serve as an independent prognosis factor for gastric cancer patients.

**Table 2:** Univariate and multivariate analysis in gastric cancer patients

Indicators	Univariate		Multivariate	
	HR (95%CI)	*p*	HR (95%CI)	*p*
Age (< 56/≥ 56)	0.62 (0.14–2.69)	0.523	NA	NA
Gender (male/female)	1.71 (0.22–13.51)	0.611	NA	NA
Differentiation (well, moderate/poor)	0.82 (0.46–1.46)	0.499	NA	NA
LN metastasis (yes/no)	2.23 (1.20–4.14)	0.011	1.98 (1.09–3.60)	0.025
UICC stage (III-IV/I-II)	2.09 (1.20–3.63)	0.009	1.59 (0.84–4.16)	0.125
SRPK1 (positive/negative)	2.23 (1.49–3.38)	< 0.000	2.05 (1.22–3.79)	0.008
IGF1R (positive/negative)	2.31 (1.51–3.45)	< 0.000	2.11 (1.19–3.82)	0.011

Note: NA = not available.

**Figure 2:** Correlations between SRPK1, IGF1R expression and prognosis of gastric cancer patients Kaplan-Meier curves curves are made for 90 gastric cancer patients with different levels of SRPK1 and IGF1R expression. (**A**) The overall survival analysis in 75 patients (high SRPK1 level) and 15 patients (low SRPK1 level). The difference between these two groups is significant based on the log-rank test. (**B**) The overall survival analysis in 78 patient (high IGF1R level) and 12 patients (low IGF1R level). The difference between these two groups is significant based on the log-rank test. High SRPK1 and IGF1R expression was obviously associated with five years prognosis of gastric cancer patients.

### The expression of SRPK1 mRNA and protein in GC cells

In an attempt to figure out the expression status of SRPK1 mRNA and protein in GC cells, including MGC803, BGC823 and HGC27 cell lines, were analyzed and tested by using RT-PCR and western blot assays, when compared with those in HC-a cells. RT-PCR assay revealed that the expression of SRPK1 mRNA was approximately 5-fold higher in MGC803, BGC823and HGC27cellsthat that in GES-1 cells (*p* < 0.001) (Figure 3A). It should be noted that the mRNA expression of SRPK1 in MGC803, BGC823 and HGC27 cells showed no significant differences (*p* > 0.05). Consistent with RT-PCR results, western blot assay revealed that the protein expression of SRPK1 was obviously higher in MGC803, BGC823 and HGC27 cells that the protein expression of SRPK1 in GES-1 cells (*p* < 0.001) (Figure 3B). At the same time, the protein expression level of SRPK1 in MGC803, BGC823 and HGC27 cells showed no significant differences (*p* > 0.05). These data indicated that the mRNA and protein expression of SRPK1 was altered in the development of GC cells.

**Figure 3:** Analysis of SRPK1 expression in GC cell lines (**A**) RT-PCR analysis of SRPK1mRNA expression in GES-1, MGC803, BGC823 and HGC27 cells. Quantification analysis was defined as the relative density of SRPK1 mRNA to GAPDH. GAPDH was used as an internal control. Results shown are the mean±SEM of repeated independent experiments. *p < 0.001, compared with control, one-way ANOVA. (**B**) The expression of SRPK1 protein was examined in GES-1, MGC803, BGC823 and HGC27cells using western blot. The average SRPK1 protein expression was normalized to β-actin. Results shown are the mean ± SEM of repeated independent experiments. *p < 0.001, compared with control, one-way ANOVA.

### The expression of IGF1R mRNA and protein in GC cells

In an attempt to figure out the expression status of IGF1R mRNA and protein in GC cells, including MGC803, BGC823 and L3252 cell lines, were analyzed and tested by using RT-PCR and western blot assays, when compared with those in GES-1 cells. RT-PCR assay revealed that the expression of IGF1R mRNA was approximately 5-fold higher in MGC803, BGC823and HGC27 cells that that in GES-1 cells (*p* < 0.001) (Figure 4A). It should be noted that the mRNA expression of IGF1R in MGC803, BGC823 and HGC27 cells revealed no significant differences (*p* > 0.05). Consistent with RT-PCR results, western blot assay revealed that the protein expression of IGF1R was obviously higher in MGC803, BGC823 and HGC27 cells that the protein expression of IGF1R in GES-1 cells (*p* < 0.001) (Figure 4B). At the same time, the protein expression level of IGF1R in MGC803, BGC823 and HGC27 cells revealed no significant differences (*p* > 0.05). These data indicated that the mRNA and protein expression of IGF1R was altered in the development of GC cells.

**Figure 4:** Analysis of IGF1R expression in GC cells (**A**) RT-PCR analysis of IGF1RmRNA expression in GES-1, MGC803, BGC823 and HGC27 cells. Quantification analysis was defined as the relative density of IGF1R mRNA to GAPDH. GAPDH was used as an internal control. Results shown are the mean±SEM of repeated independent experiments. *p < 0.001, compared with control, one-way ANOVA. (**B**) The expression of IGF1R protein was examined in GES-1, MGC803, BGC823 and HGC27cells using western blot. The average IGF1Rprotein expression was normalized to β-actin. Results shown are the mean±SEM of repeated independent experiments. *p < 0.001, compared with control, one-way ANOVA.

### IGF-1 induces SRPK1, p-AKT and EMT markers in MGC803 and BGC823 cells

To figure out the role of IGF-1 in EMT of GC, our team analyzed and detected the IGF-1-induced downstream signaling molecules and EMT biomarkers by using MGC803 and BGC823 cells and western blotting. MGC803 and BGC823 cells were treated using gradient concentrations of IGF-1 for 12 hours. By using the western blot assay, our team demonstrated and identified that the phosphorylation level of AKT and the expression level of SRPK1was obviously increased (Figure 5). In addition, we analyzed and tested the expression level of different EMT biomarkers to identify the progression of EMT. Results from western blot assay revealed thatIGF-1 can induce an obvious up-regulation of N-cadherin, MMP2 and Slug in a dose-dependent manner (Figure 5). It should be noted that the protein expression level of MMP2 is obviously enhanced, and these results suggesting that SRPK1 has a potential role in regulation of cancer cell migration and invasion.

**Figure 5:** IGF-1 induces the expression of p-AKT and EMT in MGC803 and BGC823 cells MGC803 (**A**) and BGC823 (**B**) cells were inoculated with serum-free DMEM overnight, and then complemented with gradient concentrations of IGF-1 (0, 10, 20, and 30 ng/ml). After 12 hours treatment, we conducted western blot to test the expression of corresponding proteins. This experiment was repeated three times. β-actin acts as an intern control. Each bar represents the mean ± SEM of three independent experiments; *p < 0.001, compared with control, using one-way ANOVA followed by the Dunnett *t*-test multiple comparisons test for between-group analysis.

### Knockdown of SRPK1 abrogates IGF-1-meditated EMT in MGC803 and BGC823 cells

In order to further characterize the important role of SRPK1 in the development of EMT, we knocked down the protein expression of SRPK1, and then conducted the silencing of SRPK1 using gene silencing to investigate the important role of SRPK1 on IGF-1-induced EMT. Western blot assay testified that the knockdown of SRPK1was established in MGC803and BGC823 cells due to the utility of SRPK1 siRNAs (si-SRPK1). After that, we treated MGC803 and BGC823 cells with 30 ng/ml of IGF-1 respectively and individually, and then the relevant protein expression can be evaluated as mentioned above. Our results demonstrated that the treatment of si-SRPK1 affected the expression of p-AKT, and then the treatment of si-SRPK1 also inhibited the expression of N-cadherin, MMP2 and Slug in comparison with those with non-transfectants (Figure 6). Additionally, our team noticed that the protein expression of MMP2 was seriously affected, which suggested that si-SRPK1 has an inhibitory effect on the cell migration and invasion.

**Figure 6:** Knockdown of SRPK1 abrogates IGF-1-meditated EMT in MGC803 and BGC823 cells MGC803 (**A**) and BGC823 (**B**) cells were pre-treated with si-control or si-SRPK1, and then treated as delineated above. After 12 hours incubation, western blot was used to detect the expression of corresponding proteins. The experiment was repeated three times. β-actin acts as an intern control. Each bar represents the mean ± SEM of three independent experiments; *p < 0.001, compared with control, using one-way ANOVA followed by the Dunnett *t*-test multiple comparisons test for between-group analysis.

### si-SRPK1 inhibited the cell cycle, migration and invasion

According to the data as mentioned above, our team continued to investigate the potential effect of SRPK1onthe cell cycle based on the flow cytometry, and we demonstrated that the treatment of si-SRPK1 affected G1/G0 phase entry into S phase of MGC803 and BGC823 cells (Figure 7A). After that, we further figured out the potential role of si-SRPK1 on the cell migration and invasion of MGC803 and BGC823 cells, and then we carried out the transwell assay in the present study. By way of migration assay, our results identified that knockdown of protein expression of SRPK1 affected the migratory capacity of MGC803 and BGC823 cells using wound-healing assays (Figure 7B), On the other hand, MGC803 and BGC823 cells in control group showed normal migration capacity (*p* < 0.001). By way of invasion assay, we observed that knockdown of protein expression of SRPK1 affected the invasive capacity of MGC803 and BGC823 cells in comparison with control (Figure 7C) (*p* < 0.001).

**Figure 7:** SRPK1 affects cell cycle, migration and invasion of MGC803 and BGC823 cells Cells were taken after 12 hours treatment, and DNA content was detected by flow cytometry and PI staining (**A**). The percentages of cells in the different phase are indicated. (**B**) Wound healing assay performed with MGC803 and BGC823 cells over 48 h. Cells and wounds were pretreated as described above. Wound healing within the scrape line was recorded every day. Representative scrape lines are shown at day 3; dashed line indicates the margin of the scratch at day 1. (**C**) Transwell invasion assays for cells transfected with si-SRPK1 or si-control. Each bar represents the mean ± SEM of three independent experiments; *p < 0.001, compared with control, using one-way ANOVA followed by the Dunnett *t*-test multiple comparisons test for between-group analysis.

## DISCUSSION

To date, the important role of IGF-1-SRPK1 pathway in the tumorigenesis had been widely reported, and the IGF-1-SRPK1 pathway was highly activated in a couple of tumors [12, 13]. At the same time, the gene and protein of SRPK1 are also identified to mediate the signaling pathways of tumor development [9, 10]. In the present study, we selected and demonstrated GC as study objects. Owing to malignancy of GC, it is not possible to finish the diagnosis and operation in the early stage. So, it is essential to demonstrate the important role of IGF-1-SRPK1 pathway in the development of GC cells, by which we had the chance to develop the target drugs to affect the malignant progression of GC. In the present study, some in-vitro assays were used to investigate the probable mechanisms underlying IGF-1-induced EMT of GC cells. At the beginning, we identified the SRPK1proteincan be expressed and found in GC cells. These findings suggested that SRPK1 plays an important role in the development of GC cells.

Based on the previous studies, EMT acts as a trigger which can cause the malignant transformation of normal tissue cells. After the malignant transformation, normal epithelial cells can develop into the malignant tumor cells [14]. EMT including some features due to some potential alterations of normal cell phenotype, which includes loose cell-to-cell linkage, cell motility, and invasion [15, 16]. EMT-related signaling molecules play a critical role in embryonic development, postnatal growth, and epithelial homeostasis, and then EMT is implicated in a number of pathological changes [17]. In the present study, our team selected the activator IGF-1 to induce the potential EMT pathway, and then we found the level of phosphorylated AKT and the expression of p-SRPK1were obviously enhanced and changed. Additionally, the treatment of IGF-1 also enhanced the expression of EMT biomarkers, such as the expression of N-cadherin, MMP2 and Slug in a dose-dependent fashion, which indicated that IGF-1 has a regulatory effect on EMT of GC.

After that, we further carried out the gene silencing assays to identify the actual role of IGF-1-SRPK1 pathway in EMT progression. In the recent study, van Roosmalen *et al* demonstrated that the expression of SRPK1 was correlated with metastasis of breast cancer into the lung and brain tissues [18], and then knockdown of SRPK1 seemed to repress metastasis of breast cancer into lung and brain tissues, indicating that SRPK1 plays an important role in cancer cell migration and invasion. In addition, Lin *et al* also found that SRPK1 might exert tumourigenic effects on breast cancer through RNA-binding motif protein 4-induced reduction of pro-apoptotic *IR-B* and *MCL-1S* transcripts, thereby regulating cell sensitivity to apoptotic signals [19]. Mechanically, some reports demonstrated that SRPK1 induced a stem cell-like phenotype of NSCLC probably via SRPK1-induced Wnt-β-catenin signaling [20, 21]. Overall, it is reasonable that SRPK1 induced various downstream pathways in different types of cancers, thereby leading to different cellular processes.

Taken together, our study identified the important role of SRPK1 in regulating EMT of GC. IGF-1 signaling induced the expression of SRPK1 to control the progression of EMT in the progression of GC. Our findings lay a promising foundation for the SRPK1-targeting therapy of GC patients.

## MATERIALS AND METHODS

### Ethics statement

Ethical approval was obtained from the Institutional Ethics Committee at the Ethics Committee of Shandong Provincial Third Hospital. Patients or Animals enrolled in this study signed written informed consent. All procedures were subjected to the Declaration of Helsinki.

### Patients and tissues

We included 90 cases of gastric cancer patients, including 60 men and 30 women, from Feb 2015 to Nov 2016, who underwent curative gastrectomy with lymphadenectomy at the Shandong Provincial Third Hospital. Among those patients, the average age was 56 years old (range: 45 to 72 years old). In our study, we would exclude the patients who underwent radiation therapy or chemotherapy before operation. Besides, 55 cases of adjacent normal tissues were also harvested at 5 cm away from the edge of cancer tissues. Among these tissues, 29 well differentiated, 30 moderately differentiated, and 31 poorly differentiated tissues were distinguished. Prior to our scientific research, patient's consent was obtained from the Institute Research Ethics Committee of Shandong Provincial Third Hospital. Grading of gastric cancer tissues was based on the International Union against Cancer (UICC). Eventually, follow-up databases of gastric cancer patients were obtained by a family visit or telephone. In the present study, mean follow-up time was 25 months (range: 2 to 60 months).

### Cell culture and reagents

GES-1, an immortalized human gastric epithelial cell line, was also purchased from ATCC, and cells (passages 5–10) were maintained in Gibco RPMI-1640 (Thermo Fisher Scientific, Inc.) medium supplemented with 10% FBS, 2 mM L-glutamine (Gibco; Thermo Fisher Scientific, Inc.), 100 U/ml penicillin and 100 mg/ml streptomycin. The human gastric cancer cell lineMGC803, BGC823and HGC27 were obtained from American Type Culture Collection (ATCC, Manassas, Va.), and was cultured in DMEM (Gibco) supplemented with 10% fetal bovine serum (FBS; Hyclone) and 100 U/mL penicillin/streptomycin (Gibco) and were maintained in a humidified atmosphere with 5% CO_2_ at 37°C. All experiments were performed in the absence of FBS. Recombinant human IGF-1 was obtained from Sigma Corporation (St. Louis, USA). All antibodies in this experiment can be purchased from Santa Cruz Biotechnology (Santa Cruz, USA), involving anti-p-AKT, anti-t-AKT, anti-SRPK1 (Santa Cruz Biotechnology Cat. number sc-289; 1:200); anti-N-cadherin,anti-MMP2,anti-Slug, and anti-β-actin. All assays were repeated three times.

### Immunohistochemistry

All sections were dewaxed in xylene and rehydrated in graded ethanol, followed by incubating in 3% hydrogen peroxide for 10 min to quench endogenous peroxides. Samples were heated in 0.01 mol/L citrate buffer for 15 min at 100°C, and then put at room temperature for 30 min. After cooled, samples were blocked with 2% normal goat serum in PBS for 30 min to block antigenic epitopes, and then incubated with primary antibody (1:100 dilution, Santa Cruz Biotechnology, USA) at 4°C overnight. After that, the sections were washed with PBS for three times, and then incubated with system-labeled HRP anti-mouse secondary antibody (Dako, Denmark) at room temperature for 20 minutes. Next, the sections were incubated in DAB and counterstained in Mayer's hematoxylin, dehydrated in alcohol and xylene. PBS was used as negative control. Under the microscope, the positive areas seem like brown yellow granules.

### Evaluation of immunohistochemistry staining

The score of the immunohistochemistry staining was evaluated by one investigator who was blinded to this study. And the sections were scored based on the positive percentage and staining intensity. Sections were defined as positive if there were brown yellow platy or granules in the plasma of the cells. The intensity of plasma staining was scored and graded by four scales: 0 (0% cells); 1 (0–25% cells); 2 (25–50% cells); and 3 (> 50% cells). Staining intensity was also evaluated semi-quantitatively as reported: 0 (none), 1 (mild), 2 (moderate), 3 (intense) [12]. The total score for each section was then evaluated by multiplying the intensity score and positive percentage score, and was classified into four levels: 0 (−), 1–3 (+), 4–6 (++), and 7–9 (+++). It was considered negative or low expression when the total score was less than 4.

### SRPK1 siRNA transfection

Cell lines were seeded in a 6-cm dish at density of 5×10^5^ cells/dish and incubated overnight. Twenty-four hours later, cells were prepared for transfection of SRPK1siRNA. 1 mg of SRPK1siRNA (Santa Cruz) was added to Opti-MEM with Lipofectamine 2000 (Invitrogen) for transfection, according to the manufacturer's instructions. 12 h following incubation, medium was changed into fresh DMEM containing 10% FBS. Cells were harvested at72 h following transfection of SRPK1 siRNA. Then cells were subjected to other assays.

### RNA purification, reverse transcription, and real-time PCR amplification

Total RNA was isolated 36 h after treatment with NVP-BKM120 using high pure RNA Isolation Kit (Roche). The reverse transcription (RT) reaction was performed using the revertAid First Strand cDNA Synthesis Kit (Takara BIO). The cDNA prepared was subjected to qRT-PCR on a light cycler instrument (Roche). Thermal cycling conditions included activation step for 30 s at 95°C followed by 45 cycles, including a denaturation step for 5 s at 95°C and a combined annealing/extension step for 20 s at 60°C. A melting curve analysis was applied to verify the specificity of the products, and the values for the relative quantification were calculated based on 2-ΔΔCt relative expression formula.

### Western blot analysis

Cells were centrifuged at 24 h after treatments, and cellular pellets were washed with cold PBS and lysed in RIPA buffer containing protease and phosphatase inhibitor cocktails (Sigma). After determination of protein concentrations according to Bradford method, equivalent amounts of total cellular protein were separated by 10% SDS-PAGE, and subsequently transferred to nitrocellulose membrane using a semidry transfer cell (Bio-Rad). The proteins were detected using specific primary antibodies and the enhanced chemiluminescence detection system according to the manufacturer's protocol. Band intensity was calculated using ImageJ software and the ratio of proteins to actin expression was normalized.

### Flow cytometry

Cells were detached with EDTA-free trypsin and washed with phosphate buffer saline (PBS) twice. The cells were harvested (1–5 × 10^5^). The binding buffer (50 μL) was mixed with 7-amino-actinomycin D (7-ADD) solution, and the cells were added to the mixture, followed by incubation at room temperature in the dark for 5–15 min. Flow cytometry was done by using annexin V-PE apoptosis detection kit (Invitrogen, Beijing, China) at the FL2 channel. At the excitation wavelength of 488 nm and the emission wavelength of 578 nm, orange fluorescence was observed. The 7-ADD was detected via the FL3 channel. Red fluorescence was observed at the excitation wavelength of 546 nm and emission wavelength of 647 nm. All groups were performed in triplicate.

### Wound-healing assay

Cells were placed in a 24-well plate at an initial density of 1 × 10^5^. A uniform monolayer formed in 2–3 days. All wound-healing assays were performed in a serum-free medium. A micropipette tip was used to create a wound in the monolayer by scraping. The relative cell-free area was calculated based on the control group.

### Transwell invasion assay

Transwell invasion assay was carried out using invasion chambers (Becton, Dickinson and Company, USA) pre-coated with Matrigel. Cells (2.0×10^5^/well) were seeded in the upper chamber, and medium containing CCL20 was placed into the lower chamber. After 48 h of incubation at 37°C in 5% CO_2_, noninvasive cells were removed from the upper surface of the transwell membrane with a cotton swab, and the invaded cells on the lower layer surface were fixed, stained, photographed, and counted under high-power magnification (×200).

### Statistical analysis

All data in this study were statistically analyzed using the SPSS statistical package (version 11.0 for Windows, SPSS Inc, IL, USA). Continuous variables were expressed as mean±S.D.. Differences of kindlin protein expression between osteosarcoma and corresponding noncancerous bone tissues were evaluated by the paired t test. Associations between various clinicopathological characteristics and kindlin protein expression were analyzed by X^2^ tests. Survival analyses were performed using the Kaplan-Meier and the log-rank tests. Differences were considered statistically significant when P was less than 0.05.
